The article "Implementation of Real-Time Medical and Health Data Mining System Based on Machine Learning" was published in 2021. Journal: J Healthc Eng.

# Implementation of Real-Time Medical and Health Data Mining System Based on Machine Learning

**DOI:** 10.1155/2021/7011205

**Published:** 2021-11-19

**Authors:** Pengyuan Wang, Jie Li

**Affiliations:** ^1^Zhengzhou University of Light Industry, Engineering Training Center, Zhengzhou 450001, Henan, China; ^2^The Second Affiliated Hospital of Zhengzhou University, Radiology Department, Zhengzhou 450000, Henan, China

## Abstract

This article analyzes the application process of data mining technology in the medical and health management system and uses machine learning algorithms to design a medical and health data mining system. The system collects patient's physical health data based on wireless sensing technology and uses machine learning algorithms to analyze the data. The system uploads the collected health data to the system for cluster analysis. Finally, the method is applied to the diagnosis data mining of patients, so as to prove the effectiveness of the classification method in the medical field through examples.

## 1. Introduction

Today's medical institutions have divided a wide range of specialized departments in order to provide targeted treatment. The finer the division of departments, the larger the organization of the hospital. The documentation used to record various types of medical information has also doubled [1]. This has led to a substantial increase in the difficulty and cost of managing the hospital. Therefore, it is an inevitable trend to carry out information management in hospitals.

The Internet of Things (IoT) perceives information in the physical world through wireless sensors. As an important application field of the Internet of Things, smart medical care needs to realize multidirectional information flow interaction between patients, medical staff, medical institutions, and medical equipment and expand the scope of traditional medical areas from hospitals to patients' homes [2]. Intelligently analyze the massive data streams in high-performance servers and databases in the medical Internet of Things by optimizing data processing algorithms. This can improve the effectiveness of medical services.

This paper proposes a smart medical system based on the machine learning density clustering data analysis method. Patients can use convenient high-speed broadband wireless access to the network and use smart wireless sensors to upload disease information. As the core function of the system, data-assisted analysis uses the massive data collected to make intelligent diagnosis for patients. This paper introduces a data analysis machine learning method based on the density-based spatial clustering with noise (DBSCAN) algorithm [3]. The nonlinear mapping is used to transform the patient's condition data input space into a high-latitude feature space. The DBSCAN algorithm is extended in this feature space to improve the clustering results.

The article "Implementation of Real-Time Medical and Health Data Mining System Based on Machine Learning" was published in 2021. Journal: J Healthc Eng.

### 1.1. System Design Ideas

The system is divided into three parts in terms of function. The content includes patient data collection, multiplatform login interaction, and server data processing.

Part of the patient data collection system can use wireless sensors installed on the patient to achieve ubiquitous patient physiological information collection [4]. It can provide the detection function of blood pressure, body temperature, pulse, and many other physiological indicators of the human body. And it can easily access the medical Internet of Things.

The multiplatform login interaction part adopts the B/S (browser/server) architecture. It is suitable for multiple platforms and can log in to the system at any time and anywhere through a browser.

The server data processing part is affected by the environment in the actual measurement, which inevitably generates abnormal data. Therefore, we need to adopt a data analysis algorithm that is in line with medical practice and can eliminate abnormal data. According to the above system functions, we can design the network architecture of the system (Figure 1).

## 2. Related Core Technologies

### 2.1. Hierarchical Smart Medical System Architecture

Smart medical care is an important application field of wireless sensor networks, which are wireless sensor networks with networking capabilities [5]. The system can make a large number of medical monitoring work wireless, remote, and self-service.

### 2.2. B/S and SSH Framework

The multiplatform B/S architecture refers to the browser/server architecture. The main transaction logic is implemented on the server side. SSH framework refers to the combined framework of Struts 2 + Spring + Hibernate. It is currently the most mature lightweight framework for web applications [6]. This system uses JSP technology to develop the front end, which provides a solution for creating web pages that display dynamic content.

### 2.3. DBSCAN Algorithm

There are abnormal points in the massive data entering the server, so we need to find out through data mining methods. The definition of anomalous point in the field of statistical research is as follows: based on a certain measure, the data point is significantly different from other data in the dataset.

In smart medical care, wireless sensor nodes attached to patients can perceive the measurement values of multidimensional attributes. The vector composed of the sensory measurement values of these multidimensional attributes represents the characteristic points of the patient's current physiological condition [7]. The clustering algorithm can effectively find the abnormal points of the feature points and analyze the similar data groups.

The article "Implementation of Real-Time Medical and Health Data Mining System Based on Machine Learning" was published in 2021. Journal: J Healthc Eng.

The DBSCAN algorithm is a density-based clustering algorithm. It can divide regions with sufficiently high density into clusters and find clusters of arbitrary shapes in a noisy spatial database. The algorithm finds abnormal points by ensuring that a single abnormal point does not generate a cluster. There are two parameters to control the generation of the cluster: MinPts is the minimum number of nodes in the cluster. *e* is the radius of the cluster [8]. For each point in the cluster, there must be another point in the cluster, and the distance between them is less than a certain threshold. The DBSCAN algorithm does not perform any preprocessing when operating on the data, and its time complexity is *O*(nlgn).

The local clusters of partition *SC*_1_,…, *SC*_*J*_,…, *SC*_*n*_ are merged. Any data object *p* in the overlapping zone has been clustered twice. The merging of clusters needs to be based on the information of the two clusters. *p* belongs to cluster class *A* and cluster class *B* in two adjacent overlapping partitions. If *p* belongs to the core object of class *A* or class *B* or is a core object in both classes, then class *A* and class *B* are merged into one cluster. If *p* belongs to the boundary point in both classes, then it cannot be determined that class *A* and class *B* are merged. *p* can be divided into either of the two clusters. If *p* belongs to one of these classes and is classified as a noise point in another cluster, then *p* belongs to its cluster. If *p* is classified as a noise point in the two clusters, then *p* is a noise point in the entire *D*_*i*_ partition.

Partition *D*_1_, *D*_2_,…, *D*_*i*_,…, *D*_*n*_ clusters are merged. After step 1, the internal clustering of data partition *D*_*i*_ has been completed. Since there are no overlapping partitions between partitions *D*_*i*_ and *D*_*i*+1_, the objects at the boundary of the two partitions cannot determine whether to form a cluster through the same data object. Clustering can only be done with approximate conditions based on the information of the boundary local classes (core objects, representative points, boundary positions, etc.). The clustering and merging are divided into 3 situations.

Class *CA* and class *CB* are in *D*_*i*_ and *D*_*i*+1_, respectively. The conditions that are needed to merge the classes are as follows: the Eps values of *D*_*i*_ and *D*_*i*+1_ are Eps_*i*_ and Eps_*i*+1_, Eps_min_=min(Eps_*i*_, Eps_*i*+1_),  and *E*_*A*_ and *E*_*B*_ are the set of boundary objects saved in step (1). Dist{*p*, *q*}(∀*p* ∈ *E*_*A*_, ∀*q* ∈ *E*_*B*_) is the distance of any object in the two object sets. It satisfies the following condition:

(1) $$\begin{array}{c} \bar{\text{dist}1}=\frac{\sum_{i}\sum_{j}\text{Dist}\left\{p_{i},q_{j}\right\}}{\left|E_{A}\right|*\left|E_{B}\right|}\leq {\text{Eps}}_{\min}. \end{array}$$

The noise points are merged into classes: the noise points near the boundary of *D*_*i*_ may be the boundary points of a certain class in the overall cluster. If point *p* is a noise point on the boundary of *D*_*i*_, class *C* is the class near the boundary in *D*_*i*+1_. The neighbourhood radius is Eps_*i*+1_, *E*_*c*_ is the boundary point domain set (∀*q* ∈ *E*_*c*_) saved by the class *C*. When formula (2) is satisfied, the noise point *p* is merged into the class *C*.

(2) $$\begin{array}{c} \bar{\text{dist}2}=\frac{\sum_{j}\text{Dist}\left\{p,q_{j}\right\}}{\left|E_{c}\right|}\leq {\text{Eps}}_{i+1}. \end{array}$$

Noise points are combined to form a new class: although the preprocessing of the data is based on the data distribution characteristics, there is still the possibility of dividing the same sparse cluster into different partitions to form noise points [9].

The article "Implementation of Real-Time Medical and Health Data Mining System Based on Machine Learning" was published in 2021. Journal: J Healthc Eng.

## 3. Smart Medical Management System Model

### 3.1. System User Identity Design

The users of the system are mainly medical personnel, including doctors, nurses, and equipment managers of medical units. Medical staff of any type can log in to the management system through a browser on multiple platforms. The operations that the personnel can complete are also different depending on the identity.

### 3.2. System Frame Design

#### 3.2.1. The Design of the Database

In the development phase of the system, we use MySQL database as the system database. Based on the characteristics of the ward information management system of the Internet of Things, each entity class we designed corresponds to a table. Each table has an association relationship.  Figure 2 shows the data relationship model diagram of the main table.

This system uses the data analysis method of DBSCAN algorithm. According to the characteristics of the algorithm, in addition to the general attributes, it is necessary to add data acquisition time and coordinate information for positioning [10]. The purpose of introducing coordinate information is to facilitate the conversion of a single data value into a data point in space. Its value is set to be equivalent to the obtained body data information.

#### 3.2.2. The Design of the Front Page

According to different job permissions, the front page is divided into patient page, doctor page, nurse page, and administrator page. Each page has functional modules to complete the corresponding duties. Different positions display different interfaces. When the corresponding ordinary post performs a higher authority operation, the system goes to the failure page and prompts that the authority is insufficient.

The article "Implementation of Real-Time Medical and Health Data Mining System Based on Machine Learning" was published in 2021. Journal: J Healthc Eng.

#### 3.2.3. The Design of the Back-End Server

The background server part uses Tomcat as the web server. Tomcat is an open-source web application server. It occupies small system resources during operation, has good scalability, and supports common functions of development application systems such as load balancing and mail service.

### 3.3. Data Analysis of the DBSCAN Algorithm

Another core part of the system is data analysis and research. The design idea is to use the DBSCAN algorithm to process the data to obtain different data clusters [11]. Then, the cluster is compared with the standard data to make a judgment. In the system, data are collected by sensors and smart medical equipment and then uploaded to the database server. Algorithm wisdom is used to eliminate abnormal data, and then the useful data are analyzed to get the result. The whole process is shown in Figure 3.

Data analysis of patients' blood pressure, body temperature, etc., needs to be analyzed after removing abnormal points. We use the DBSCAN algorithm to process patient blood pressure, body temperature, and other data. The article divides the data into categories. Those isolated few points will be regarded as abnormal points and eliminated, and the remaining data clusters will be regarded as useful data. The DBSCAN algorithm has 3 important definitions, which, respectively, explain the concepts of density reachability, density connection, and clusters.

The data cluster retained by the system is the true embodiment of the patient's physiological data. These data are used for comparison with standard health data. The cause of the disease can be judged according to the deviation value of various physiological data; that is, the intelligent diagnosis of the system is completed.

This data analysis method has strong flexibility. The parameters of the algorithm can be changed according to the patient's symptoms. For patients with severe disease, the number of measurements can be increased, the size of MinPts can be increased, and the value of *ε* can be reduced [12]. In this way, the patient's current physiological data can be obtained more accurately. Patients with certain chronic diseases can extend the length of time period selection and increase the number of time periods selected. Using the algorithm multiple times can get the patient's physiological condition over a long period of time and make a smart diagnosis.

The article "Implementation of Real-Time Medical and Health Data Mining System Based on Machine Learning" was published in 2021. Journal: J Healthc Eng.

## 4. Experimental Results

This article uses MATLAB to write functional programs. We choose the actual data obtained by a third-class general hospital for verification. The article collects statistics of the detection data obtained by a certain department of the hospital using physiological information detection equipment similar to this system within half a year to form an independent database. Then, the DBSCAN algorithm is used for processing and analysis. The physiological information feature extraction data before the diagnosis and the diagnosis conclusion after the diagnosis are bound for processing. In this way, the accuracy of the forecasting ability can be improved.

Table 1 shows the comparison between actual data and predicted data of comprehensive physiological characteristic values. It can be obtained that the error between the predicted data and the actual data is 5.5%. This shows that the results of the predictive model are close to reality.

## 5. Concluding Remarks

The intelligent medical information system is an important part of the current medical development. This paper proposes a data analysis method of the DBSCAN deep learning algorithm based on the wireless sensor technology of the Internet of Things to collect patient physiological information data. The algorithm can eliminate abnormal data and cluster valid data. Comparing clustered data with health data can make a judgment on the cause of the disease. Based on this, it can be concluded that the results of smart diagnosis can effectively provide medical staff with reference for treatment.

## Figures and Tables

**Figure 1:** Smart medical system architecture.

**Figure 2:** Data relationship diagram.

**Figure 3:** Data processing flow.

**Table 1:** Comprehensive physiological characteristic values.

Serial number	Nominal value	Predictive value	Error (%)
1	3.1	3.16	1.9
2	3.4	3.22	5.3
3	2.9	3.10	6.5
4	3.4	3.26	4.1
5	2.8	3.10	10.7
6	2.9	2.87	1.0
7	2.7	2.84	5.2
8	2.8	3.01	7.5
9	2.8	2.97	6.1
10	2.6	2.77	6.5

## Data Availability

The data used to support the findings of this study are available from the corresponding author upon request.
